# Efficacy and Mechanism of Trimebutine Maleate Combined with Lactulose in the Treatment of Constipation-Predominant Irritable Bowel Syndrome in the Elderly

**DOI:** 10.1155/2022/6125120

**Published:** 2022-11-11

**Authors:** Yeping Zhou, Dujuan Yang, Wenjun Gu

**Affiliations:** ^1^Department of Gastroenterology, Zhuji People's Hospital, Zhuji, Zhejiang 311800, China; ^2^Department of Geriatric, Zhuji People's Hospital, Zhuji, Zhejiang 311800, China; ^3^Department of Gastroenterology, The Ninth People's Hospital, Shanghai Jiaotong University School of Medicine, Shanghai 200011, China; ^4^Shanghai Key Laboratory of Gut Microecology and Associated Diseases, The Digestive Disease Research and Clinical Transformation Center, SJTU 200011, Shanghai, China

## Abstract

**Objective:**

Study on the efficacy and mechanism of trimebutine maleate combined with lactulose in the treatment of constipation-predominant irritable bowel syndrome (IBS-C) in the elderly.

**Methods:**

From March 2019 to March 2021, 102 elderly patients with IBS-C were randomly divided into the observation group (51 cases) and the control group (51 cases). The observation group was treated with trimebutine maleate combined with lactulose, while the control group was treated with lactulose. Comparison of the clinical effects of the two groups. Comparison of vasoactive intestinal peptide (VIP) levels, neuropeptide Y (NPY) levels, and quality of life scores before and after treatment between the two groups. Documentation of adverse reactions during treatment.

**Results:**

The improvement of clinical symptoms in the observation group was significantly better than that in the control group, and the difference is statistically significant (*P* < 0.05). The level of VIP after treatment in the observation group was significantly lower than that in the control group and before treatment, and the differences were statistically significant (*P* < 0.05). The level of NPY after treatment in the observation group was significantly higher than that in the control group and before treatment, and the differences were statistically significant (*P* < 0.05). The scores of dietary restrictions and health worries in the control group after treatment were significantly higher than those before treatment, and the differences were statistically significant (*P* < 0.05). The scores of anxious, behavioral conflict, dietary restrictions, health worries, social response, and family relationship in the observation group after treatment were significantly higher than those in the control group and before treatment, and the differences were statistically significant (*P* < 0.05). There were no serious adverse effects in either group during the treatment period, with some patients experiencing dizziness and dry mouth, which improved after discontinuation of the drug, without special intervention.

**Conclusion:**

Trimebutine maleate combined with lactulose can improve clinical symptoms and quality of life in elderly patients with IBS-C, and its mechanism of action may be related to the regulation of the body's VIP and NPY levels.

## 1. Introduction

Irritable bowel syndrome (IBS) is a nonorganic disease. Its main symptoms are functional gastrointestinal disease symptoms such as abdominal pain, abdominal distension, and abnormal defecation [1]. The protracted course of IBS has a serious impact on the quality of life of patients [2]. The pathogenesis of IBS may be related to high visceral sensitivity, intestinal infection, dysbiosis of microflora, genetics, diet, and mental factors [3, 4]. Lactulose is a synthetic disaccharide that is not absorbed by the small intestine, increases fecal water content, lowers intestinal pH, and promotes intestinal motility. It has been found that lactulose can correct and restore the intestinal microecological balance and can be used as a conventional medicine for the treatment of constipation-predominant irritable bowel syndrome (IBS-C) [5]. Trimebutine maleate is a commonly used clinical drug for the treatment of IBS, which can adjust the abnormal gastrointestinal rhythm and is suitable for the adjuvant treatment of patients with gastrointestinal dysfunction and IBS, but mostly diarrhea-type [6]. In addition, clinical reports on the combination of the two are rare, in order to clarify the clinical effect and mechanism of trimebutine maleate combined with lactulose in the treatment of IBS-C in the elderly, this clinical controlled study was conducted, and the results are reported as follows:

## 2. Materials and Methods

### 2.1. General Data

102 elderly patients with IBS-C who were admitted to our hospital from March 2019 to March 2021 were selected, and the patients were divided into the observation group (51 cases) and the control group (51 cases) by the random number table method. This study was reviewed and approved by the hospital ethics committee, and the included patients gave informed consent to this study and signed the informed consent. In the observation group, there were 25 males and 26 females, aged 60–74 years, mean age (66.42 ± 4.62) years, disease duration of 3–24 months, mean disease duration (15.23 ± 6.84) months, total symptom score of 10–17 points, with an average of (14.12 ± 3.16) points. In the control group, there were 26 males and 25 females, aged 60–75 years, mean age (67.08 ± 4.71) years, disease duration of 3–24 months, mean disease duration (15.41 ± 6.92) months, total symptom score of 10–18 points, with an average score of (15.01 ± 3.22) points. There was no significant difference in general data between the two groups (*P* > 0.05), and there was comparability.

### 2.2. Inclusion Criteria

Inclusion criteria were as follows: (1) aged 60–75 years old; (2) symptoms in the past 3 months met the diagnostic criteria of IBS Rome III [7], that is, symptoms for more than six months, abdominal discomfort or pain that has persisted for the last three months and is accompanied by at least two of the following characteristics: symptoms improve after defecation, symptoms occur with a change in the frequency of defecation, symptoms occur with a change in the nature of defecation; (3) The clinical symptoms of IBS-C are mainly incomplete bowel movements, hard lumpy bowel movements, obstructive sensation in the anus during defecation, inability to help oneself to defecation and the need for external assistance; (4) on clinical examination, gastrointestinal tumors were excluded; (5) those with complete clinical data.

### 2.3. Exclusion Criteria

Exclusion criteria were as follows: (1) patients with mental disorders; (2) patients unable to communicate with normal speech; (3) patients with alarm symptoms such as anemia, blood in the stool, and weight loss; (4) patients with severe respiratory and central nervous system diseases; (5) patients with severe liver and kidney dysfunction.

### 2.4. Treatment Methods

Both groups received routine diet therapy and psychological and behavioral therapy. On these bases:

#### 2.4.1. Control Group

Routine treatment was used. That was lactulose oral solution (produced by Beijing Hanmei Pharmaceutical Co., Ltd., approved by Chinese medicine H20065730) 10∼25 ml was used, which was taken with breakfast, and the course of treatment was 12 weeks.

#### 2.4.2. Observation Group

Treatment with trimebutine maleate combined with lactulose. The dosage of lactulose was referred to as that of the control group; at the same time, it was combined with trimebutine maleate dispersible tablets (produced by Zhejiang Anglikang Pharmaceutical Co., Ltd., approved by H20040882) orally, 2 tablets (0.2 g) each time, 3 times a day, and the course of treatment was 12 weeks.

#### 2.4.3. Observation Indicators

(1) Clinical effect: collect patients' abdominal pain time, abdominal pain frequency, abdominal pain and distention during defecation, abnormal defecation character ratio, abnormal defecation frequency ratio, and mucous stool ratio to evaluate by symptom score, and count the total symptom score before and after treatment. (Symptom score before treatment - symptom score after treatment)/symptom score before treatment, the calculated value was converted into a percentage, and the clinical symptom decline rate of the patient was obtained. ≥ 90% was considered healed, 80–90% was a significant effect, 60–79% was valid, and < 60% was invalid. (2) Vasoactive intestinal peptide (VIP) and neuropeptide Y (NPY) levels: fasting cubital venous blood was collected from patients before and after treatment, and serum was collected after centrifugation. The determination was carried out by professional inspectors in strict accordance with the instructions of the inspection reagents. (3) Quality of life: the irritable bowel syndrome-quality of life (IBS-QOL) was used to evaluate, a total of 34 items, 8 dimensions, anxious, behavioral conflict, body image, dietary restrictions, health worries, social response, sexuality, and family relationship were scored on a 5-point scale, namely, asymptomatic, mild, moderate, severe, and severe were scored as 5, 4, 3, 2, and 1, respectively, and the scores of each dimension were converted into percentage values (the actual score/full score of each dimension × 100%) for statistics, the higher the score, the better the quality of life. (4) Documentation of adverse reactions during treatment.

### 2.5. Statistical Methods

Data were entered into Excel form, imported into SPSS24.0 for statistical processing, measurement data were expressed as mean ± standard deviation (*x* ± *s*), and a *t*-test was applied; The enumeration data were expressed by the rate (%), and the *χ*^2^ test was used. The rank data was expressed by the rank sum test, and there was a significant difference at *P* < 0.05.

## 3. Results

### 3.1. Clinical efficacy of patients

The improvement of clinical symptoms in the observation group was significantly better than that in the control group, and the difference is statistically significant (*P* < 0.05) (as shown in Table 1).

### 3.2. Comparison of VIP and NPY Levels in Patients

Before treatment, there was no significant difference in the levels of VIP and NPY between the two groups (*P* > 0.05); The level of VIP after treatment in the observation group was significantly lower than that in the control group and before treatment, and the differences were statistically significant (*P* < 0.05). The level of NPY after treatment in the observation group was significantly higher than that in the control group and before treatment, and the differences were statistically significant (*P* < 0.05) (as shown in Table 2).

### 3.3. Comparison of Patients' Quality of Life

There was no significant difference in the scores of each dimension of the IBS-QOL scale between the two groups before treatment (*P* > 0.05); The scores of dietary restrictions and health worries in the control group after treatment were significantly higher than those before treatment, and the differences were statistically significant (*P* < 0.05). The scores of anxious, behavioral conflict, dietary restrictions, health worries, social response, and family relationship in the observation group after treatment were significantly higher than those in the control group and before treatment, and the differences were statistically significant (*P* < 0.05) (as shown in Figure 1).

### 3.4. Documentation of Adverse Reactions during Treatment

There were no serious adverse effects in either group during the treatment period, with some patients experiencing dizziness and dry mouth, which improved after discontinuation of the drug, without special intervention.

## 4. Discussions

The incidence of IBS gradually increases with the change in people's life and diet structure [8]. With the in-depth study of the pathogenesis of IBS, the theories of NPY, vasoactive peptides, other gastrointestinal hormones, and abnormal visceral sensitivity have been paid more and more attention by scholars [3, 9]. NPY mainly exists in ileum and colon cells and is a biologically active substance with the function of regulating gastrointestinal motility [10]. A vasoactive peptide is a noncholinergic inhibitory gastrointestinal hormone secreted by the gastrointestinal mucosa, which can inhibit the contractile function of the smooth muscle of the gastrointestinal tract, inhibit the excitability of the gastrointestinal tract, reduce the motility of the gastrointestinal tract, cause gastrointestinal motility, and gastrointestinal emptying is impaired [11, 12]. Studies have shown that VIP acts as an inhibitor of gastrointestinal motility and that VIP is elevated in the intestinal mucosa of patients with IBS-C, resulting in an inhibitory background of intestinal motility such that peristaltic contractions are less likely to occur, leading to constipation. Based on the above, aiming at improving gastrointestinal hormone levels and reducing visceral sensitivity can more effectively improve the clinical symptoms of IBS-C patients.

Lactulose can be converted into organic acids of molecular weight with the assistance of the digestive tract flora, which helps to reduce the pH value in the intestinal tract, stimulates the smoothness of the intestinal tract, relieves constipation, and helps restore the physiological activity of the colon. It has high safety and is suitable for patients with IBS-C [13, 14]. Trimebutine maleate is a commonly used drug for patients with diarrhea-type irritable bowel syndrome and has the function of regulating gastrointestinal motility [15, 16]. Relevant data show that the effect of trimebutine maleate or lactulose alone in the treatment of elderly IBS-C is not ideal, and it has certain limitations. Therefore, this study will combine the two to observe its efficacy and explore its possible mechanism of action.

The results of this study showed that the improvement of clinical symptoms in the observation group was significantly better than that in the control group (*P* < 0.05). This indicates that trimebutine maleate combined with lactulose has a synergistic effect in the treatment of IBS-C in the elderly, with a more definite improvement in their clinical symptoms. Analyze the reasons for the above results: On the one hand, lactulose has the characteristics of disaccharide intestinal nonabsorption, can support the reproduction of intestinal bifidobacteria and lactobacilli, correct and restore the intestinal microecology, and acidic metabolites such as lactic acid and acetic acid can promote intestinal peristalsis, increase the osmotic pressure in the intestine, soften the stool and promote stool excretion. On the other hand, trimebutine maleate is gastric motility regulating drug, in addition to blocking the calcium influx channel to make gastrointestinal smooth muscle in a relaxed state, it can also effectively inhibit the outflow of potassium ions to enhance the excitability of smooth muscle cells. The main mechanism of trimebutine maleate is that it can reduce the release of acetylcholine to improve gastrointestinal motility when the gastrointestinal tract is in a highly dynamic state for a long time; in the low dynamic state, it can effectively control the release of adrenaline to improve gastrointestinal movement, thereby realizing bidirectional regulation.

At the same time, the level of VIP after treatment in the observation group was significantly lower than that in the control group and before treatment (*P* < 0.05), and the level of NPY after treatment in the observation group was significantly higher than that in the control group and before treatment (*P* < 0.05). The above shows that the treatment of trimebutine maleate combined with lactose can synergistically work together to inhibit the release of VIP and promote the release of NPY, thereby modulating visceral hypersensitivity in elderly IBS-C patients. Studies [17] have shown that elderly IBS-C patients have increased intestinal mucosal mast cell and VIP expression, and decreased NPY expression, so show high visceral sensitivity. The decrease in VIP levels was more pronounced in the observation group of this study, indicating a significant decrease in visceral sensitivity in patients, which is more helpful in improving the symptoms of visceral hypersensitivity, gastrointestinal motility disorders, and impaired gastrointestinal emptying. At the same time, trimebutine maleate can effectively inhibit the plasma substance P and somatostatin in patients, thereby promoting the release of NPY [18, 19]. Therefore, the combination of the two has the effect of inhibiting the high sensitivity of the viscera and correcting intestinal endocrine function. The observation of the quality of life of the patients showed that the improvement of the quality of life of the patients in the observation group was more significant. There were no serious adverse effects in either group during the treatment period, with some patients experiencing dizziness and dry mouth, which improved after discontinuation of the drug, without special intervention. However, due to the small sample size and short observation time included in this study, clinical large-sample studies are still needed for verification.

In conclusion, trimebutine maleate combined with lactulose can improve clinical symptoms and quality of life in elderly patients with IBS-C, and its mechanism of action may be related to the regulation of the body's VIP and NPY levels.

## Figures and Tables

**Figure 1:** Comparison of IBS-QOL scores between the two groups of patients (scores, ‾*x* ± *s*). Note: compared with the same group before treatment, ^*∗*^*P* < 0.05; compared with the control group after treatment, Δ*P* < 0.05. (a) Anxious. (b) Behavioral conflict. (c) Body image. (d) Dietary restrictions. (e) Health worries. (f) Social response. (g) Sexuality. (h) Family relationship.

**Table 1:** Comparison of clinical symptoms of patients (*n*, %).

Group	*n*	Healed	Significant effect	Valid	Invalid
Control group	51	16	20	9	6
Observation group	51	29	20	2	0
*Z*			3.234		
*P*			0.012		

**Table 2:** Comparison of VIP and NPY levels in patients (pg/ml, ‾*x* ± *s*).

Group	*n*	VIP		NPY	
		Before treatment	After treatment	Before treatment	After treatment
Control group	51	292.30 ± 47.09	242.31 ± 35.06	60.52 ± 7.94	67.17 ± 9.23
Observation group	51	294.45 ± 47.05	173.35 ± 30.07	60.22 ± 7.53	85.17 ± 9.28
*T*		0.231	10.662	0.196	9.821
*P*		0.818	0.000	0.845	0.000

## Data Availability

The data can be obtained from the author upon reasonable request.
